The article "Comparative Analysis of Different Efficient Machine Learning Methods for Fetal Health Classification" was retracted in 2023. Reasons: signs of a paper mill; compromised peer review; unreliable results or conclusions.

# Comparative Analysis of Different Efficient Machine Learning Methods for Fetal Health Classification

**DOI:** 10.1155/2022/6321884

**Published:** 2022-04-21

**Authors:** Md Takbir Alam, Md Ashibul Islam Khan, Nahian Nakiba Dola, Tahia Tazin, Mohammad Monirujjaman Khan, Amani Abdulrahman Albraikan, Faris A. Almalki

**Affiliations:** ^1^Department of Electrical and Computer Engineering, North South University, Bashundhara, Dhaka 1229, Bangladesh; ^2^Department of Computer Science, College of Computer and Information Sciences, Princess Nourah bint Abdulrahman University, P. O. Box 84428, Riyadh 11671, Saudi Arabia; ^3^Department of Computer Engineering, College of Computers and Information Technology, Taif University, P. O. Box 11099, Taif 21944, Saudi Arabia

## Abstract

Obstetricians often utilize cardiotocography (CTG) to assess a child's physical health throughout pregnancy because it gives data on the fetal heartbeat and uterine contractions, which helps identify whether the fetus is pathologic or not. Obstetricians have traditionally analyzed CTG data artificially, which takes time and is unreliable. As a result, creating a fetal health classification model is essential, as it may save not only time but also medical resources in the diagnosis process. Machine learning (ML) is currently extensively used in fields such as biology and medicine to address a variety of issues, due to its fast advancement. This research covers the findings and analyses of multiple machine learning models for fetal health classification. The method was developed using the open-access cardiotocography dataset. Although the dataset is modest, it contains some noteworthy values. The data was examined and used in a variety of ML models. For classification, random forest (RF), logistic regression, decision tree (DT), support vector classifier, voting classifier, and K-nearest neighbor were utilized. When the results are compared, it is discovered that the random forest model produces the best results. It achieves 97.51% accuracy, which is better than the previous method reported.

## 1. Introduction

In 2012, there were around 213 million pregnancies globally [1]. Pregnancy was reported in 190 million impoverished countries (89%) and 23 million developed countries (11%). In 2013, 293,336 women died as a result of pregnancy-related complications, including maternal hemorrhage, abortion difficulties, high blood pressure, maternal infection, and obstructed labor [2]. According to the World Health Organization (WHO) [3], over 303,000 women died during and after pregnancy and delivery in 2015, with approximately 830 women dying every day as a result of pregnancy or childbirth-related complications. Medical difficulties and mortality associated with pregnancy are still a major concern worldwide nowadays, affecting mothers and/or their babies. Maternal mortality is very high in many parts of the world. Indeed, impoverished countries are responsible for nearly 99 percent of maternal deaths [3]. This disproportionately large and uneven distribution of mortality reflects global disparities in access to medical care and treatment. Not just across nations, but even within countries, there are substantial variations in mortality. Even when comparing high- and low-income females, as well as rural and urban women, there are still variations in mortality. As a result, in developing countries, pregnancy and delivery problems are among the major causes of death [2, 3]. While the bulk of these problems occur during the period of pregnancy, some develop before and are worsened by pregnancy. Almost all of these maternal deaths, however, happened in resource-limited conditions, and the vast majority of them could have been avoided or cured. Pregnancy complications include hypertension, gestational diabetes, infection, preeclampsia, pregnancy loss and miscarriage, preterm labor, and still birth. Additionally, severe nausea, vomiting, and anemia due to an iron shortage are also possible [4, 5]. Thus, these illnesses may jeopardize pregnancy, necessitating the development of novel techniques for monitoring and assessing fetal well-being. These disorders may include maternal health issues that affect the infant, pregnancy-related difficulties, and fetal diseases [6]. Essential hypertension, pre-eclampsia, renal and autoimmune disease, maternal diabetes, and thyroid disease are among medical difficulties for the mother [7–10]. Prolonged pregnancy, vaginal bleeding, decreased fetal movements, and persistent ruptured membranes are other pregnancy-related medical issues that put the fetus's health at danger [11]. Furthermore, intrauterine growth restriction, fetal infection, and numerous pregnancies all put the fetus at risk [11, 12]. As a consequence, these disorders can cause neuron developmental issues throughout infancy, such as non-ambulant cerebral palsy, developmental delay, auditory and visual impairment, and fetal compromise, all of which can lead to morbidity or death in the newborn.

Cardiotocography (CTG) is a commonly used technical method for constantly monitoring and recording the fetal heart rate (FHR) and uterine contractions during pregnancy in order to evaluate fetal well-being and diagnose an increased risk of pregnancy problems. This allows the monitoring and early intervention of embryonic hypoxia before severe asphyxia or death [13]. During uterine contractions, the FHR and its variability, responsiveness, and probable decelerations are key indications of fetal well-being [14]. The FHR measurements may be taken by putting an ultrasound transducer on the mother's tummy. The CTG is utilized to discover and detect harmful abnormalities in the newborn based on the FHR, uterine contractions, and fetal movement activity. Obstetricians often use the CTG to assess and evaluate fetal status throughout the prenatal and postnatal stages of pregnancy and delivery. Recent advancements in medical technology have allowed the adoption of robust and effective ML and artificial intelligence methods to offer automated prediction in a range of medical applications based on early detection findings [15–18]. Implementing and demonstrating the suitability of ML tools can help health professionals make more informed medical decisions and diagnoses, effectively reducing maternal and fetal death rates and problems during pregnancy and childbirth, and benefiting populations in both developing and developed countries. While detecting the FHR is difficult, computer-aided detection (CAD) approaches based on ML have been designed to provide automated fetal status classifications during pregnancy [19]. For this reason, the main motivation of this paper is to implement different types of machine learning algorithms to detect fetal health-related problems in a short time. Previously, published research utilized CAD techniques to evaluate fetal health during pregnancy, specifically a support vector machine (SVM) algorithm using a Gaussian kernel function [20, 21]. Furthermore, cardiotocograms have also been categorized by neural network and random forest classifiers [22, 23].

Huang [24] used three distinct ML approaches to examine CTG data in order to predict fetal distress. The use of statistical features from empirical mode decomposition (EMD) was presented by Krupa et al. [25]. The sub-band decomposition properties were divided into two categories: normal and harmful. When it came to test data, they achieved an accuracy of 86 percent. A two-step assessment of fetal heart rate data was given in another study, allowing for accurate acidemia risk prediction. SVM, fuzzy logic, and multilayer perceptrons are used to classify the FHR signals. Sundar et al. [26] used an artificial neural network to create a new model for categorizing CTG data (ANN). To evaluate performance, the recall and F-score were utilized. They also suggested using k-means clustering to categorize CTGs [26]. Adaptive neuro-fuzzy inference techniques were utilized by Ocak and Ertunc [27] to classify CTGs (ANFIS). Ocak also developed a classification algorithm based on SVM and genetic algorithms (GA) [28]. In [29–33], the authors have used various models and algorithms for machine learning, deep learning, and others.

According to this research, ML algorithms have a substantial impact on fetal health classification. The current study is mostly focused on identifying fetal health as quickly as possible. As a consequence, fetal conditions must be detected early, requiring the use of specialized methods.

The main contribution of this study is that we applied some well-known ML techniques. Among these algorithms, the random forest, decision tree, K-nearest neighbor, voting classifier, support vector classifier, and logistic regression achieved 97.51 percent, 95.70 percent, 90.20 percent, 97.45 percent, 96.57 percent, and 96.04 percent accuracy, respectively. Also, the novelty of this research is that the accuracy percentage of the models utilized in this investigation is clearly higher than in earlier studies, indicating that the models in this study are more reliable. Multiple model comparisons have confirmed their robustness, and the scheme may be derived from the study analysis.

According to studies, the situation may improve if women can discover fetal health-related problems early and receive treatment at an early stage. They must do so by precisely predicting the progression of the disease from a moderate state to a serious fetal condition. ML technology can assist in making accurate predictions at an early stage. Many ML systems exist, but their predictions are unreliable and erroneous. They also have concerns with overfitting and underfitting. As a consequence, the main objective of this research is to develop a model to help medical technicians identify fetal illness early using ML. It will confirm and demonstrate if someone has a fetal health problem during their pregnancy.

The remainder of this work is laid out as follows. The method and experiment methodology are discussed in Section 2.  Section 3 discusses the results and analysis, and Section 4 discusses the conclusions.

## 2. Method and Materials

This section covers all methods and materials, as well as the dataset's description, block diagram, flow diagram, and evaluation matrices.

### 2.1. Dataset

This section introduces the cardiotocography (CTG) dataset's descriptions and features related pregnancy problems. The cardiotocography dataset utilized in this study was acquired from the UCI ML repository database [34]. This dataset comprises data on the FHR and uterine contraction parameters measured using cardiotocograms during pregnancy. The Biomedical Engineering Institute in Porto, Portugal, and the Faculty of Medicine at the University of Porto, Portugal, provided the data in September 2010.These datasets were acquired in 1980 and again between 1995 and 1998 on a regular basis, resulting in an ever-growing collection. This dataset includes 2126 records representing characteristics derived from cardiotocogram examinations that were then categorized into three categories by three expert obstetricians: normal, suspect, and pathological. The total amount and percentage of normal, suspect and pathological data in the fetal health classification dataset is shown in Figures 1 and 2. In the coding part, normal, suspect, and pathological are replaced as 1, 2, and 3, respectively.

Figures 1 and 2 show that the dataset is imbalanced. For this reason, the datasets have been balanced using a variety of techniques. There are no missing attributes in the dataset, and the class distribution is 1655 normal, 295 suspect, and 176 pathological.  Figure 3 shows the total number of normal, suspect, and pathological data after balancing.

Due to the dataset's imbalance, the Synthetic Minority Oversampling Technique (SMOTE) was employed to balance it [35]. SMOTE is used to prevent the ML model from being overfit on skewed classes. This method was first evaluated on training folds before being used on actual, intact, and previously unknown data.

### 2.2. Block Diagram of the System

The architectural diagram of the ML system is shown in Figure 4. The system makes use of the CTG dataset, which includes all of the characteristics and values. To begin, we examined the dataset for categorical values and found just one. This column of attributes is transformed to the numeric values 1, 2, and 3. We examined the correlations between characteristics using the “correlation matrix” function based on fetal state attributes and displayed them in order to better comprehend them.

The characteristics necessary for prediction have been assigned, and the goal value has been specified so that the model can forecast. The dataset was then separated into training and testing subsets. Although random sampling was utilized to determine the split, this results in an imbalance between the training and testing halves. As a result, stratified sampling was used with a training size of 77% and a testing size of 33%. Following that, standardization was used to scale the features. Additionally, additional histograms and scatter plot visualizations were performed on the training split to help visualize the situation. Then, the system's training started. All models were developed using the scikit-learn framework.

### 2.3. Flowcharts of the System

Fetal health is the most frequent illness diagnosed in the medical profession, and it is increasing year after year. A comparison of six widely used ML algorithms for classification fetal state recurrence is done using the CTG dataset:

- Random forest
- Decision tree
- K-nearest neighbor
- Logistic regression
- Support vector classification
- Voting classifier

#### 2.3.1. Random Forest Flowchart

The flowchart for the full random forest model is shown in Figure 5. The random forest is a machine learning technique for guided learning [36]. It constructs a “forest” from a selection of trees that have been mostly prepared for the “bagging” technique. The bagging technique is fundamentally justified since mixing several learning models enhances the final result. The random forest creates a large number of different trees and then combines them to provide a more accurate and reliable representation. It has the advantage of addressing the arrangement and relapse issues that afflict the majority of existing ML frameworks. Another notable aspect of the random forest technique is the ease with which the general significance of each component in the estimate may be determined. Sklearn has an incredible apparatus for determining an element's importance by evaluating how much pollution is decreased across the forest by the tree centers that utilize it. It then calculates this score for each brand and changes the results in order to increase their absolute importance.

The flexibility of random forest is one of its most alluring features. It may be utilized for both relapse detection and grouping tasks, and the overall weighting given to information characteristics is readily apparent. Additionally, it is a beneficial approach since the default hyper parameters it employs often give unambiguous expectations. Understanding the hyper parameters is critical, since there are relatively few of them to begin with. Overfitting is a well-known problem in ML, although it occurs seldom with the arbitrary random forest classifier. If there are sufficient trees in the forest, the classifier will not overfit the model.

The random forest method is composed of a series of decision trees, each of which is constructed using a bootstrap sample from a training set. The out-of-bag (OOB) sample, which we shall discuss later, is one-third of the training sample that is kept for testing purposes. The dataset is then injected with another instance of randomization through feature bagging, increasing its variety while decreasing the correlation across decision trees. The method for forecasting varies according to the circumstance.

#### 2.3.2. Decision Tree Flowchart

Figure 6 depicts the whole decision tree design flowchart. This study makes use of a decision tree classifier. This classifier [37] seems to recursively divide the example space. It is a predictive paradigm that acts as a mapping between the characteristics of an item and their values [38]. It regularly splits each potential data result into parts. Each nonleaf node corresponds to a feature experiment, each branch to the outcome of the experiment, and each leaf node to a judgment or classification [39]. The root node of the tree, which is at the very top, reflects the most often used prediction model. The decision node and the leaf node are the two nodes in a decision tree. The choice nodes are used to make those selections and have numerous branches, whereas the leaf nodes are the result of those choices and contain no additional branches. The outcomes of the tests or judgments are contingent on the dataset's properties.

The choice tree is easy to comprehend since it replicates the phases that a person goes through while making a real-world decision. It may be very beneficial in resolving issues with decision-making. Consider all potential solutions to an issue. Cleaning data is not required as much as it is with other methods.

#### 2.3.3. K-Nearest Neighbor

The flowchart in Figure 7 illustrates the whole K-nearest neighbor concept. The K-nearest neighbor method is a key component of ML. It is based on the technique of supervised learning. The K-NN strategy implies that the new case/data and previous cases are comparable and it assigns the new case to the category that is closest to the previous categories. The K-NN algorithm keeps all available data and categorizes new data points depending on how comparable they are to earlier classified data. This implies that fresh data may be rapidly categorized into a well-defined category using the K-NN technique. While the K-nearest neighbor (KNN) technique is applicable to both regression and classification issues, it is more often employed for classification problems. The K-NN method is nonparametric, meaning it does not make any assumptions about the data. It is sometimes referred to as a lazy learner method because it does not learn from the training set right away, instead storing and categorizing the data later. The KNN method merely saves the knowledge during the training phase, and when it receives new data, it categorizes it into a category that is very comparable to the new data.

This study uses the K-nearest neighbor classifier, which is one of the most frequently used classification algorithms in ML [38]. The K-nearest neighbor approach is a nonparametric method for classifying data. This classifier classifies objects according to their proximity and “k” closest neighbors. It is concerned with the immediate surroundings of the item rather than with the required data distribution [39].

#### 2.3.4. Logistic Regression

Figure 8 depicts the flowchart for the logistic regression model. In the supervised learning technique, the logistic regression is one of the most commonly used ML algorithms [40]. It is a forecasting technique that makes use of a group of independent variables to anticipate the value of a categorical dependent variable.

The output of a categorical dependent variable is forecasted using logistic regression. As a result, the output must be either categorical or discrete. It may be Yes or No, 0 or 1, true or false, and so on, but probabilistic values between 0 and 1 are given instead of precise values like 0 and 1. In terms of application, logistic regression and linear regression are nearly identical. Linear regression is utilized to address regression issues, whereas the logistic regression is utilized to handle classification issues. We utilize logistic regression to fit a “S”-shaped logistic function that predicts two maximum values, rather than fitting a regression line (0 or 1). The curve of the logistic function reflects the likelihood of something, such as whether cells are malignant or not, or whether a mouse is fat or not based on its weight. Because it can produce probabilities and classify new data using both continuous and discrete datasets, logistic regression is a common ML technique.

#### 2.3.5. Support Vector Machine

The support vector machines are a powerful and adaptable supervised ML approach [41]. They are used for both classification and regression. However, they are often employed in categorization issues. SVMs were introduced in the 1960s but were improved in 1990. SVMs are implemented differently than other ML algorithms. They have been very popular in recent years because of their capacity to handle a large number of continuous and categorical variables. The classification technique of the SVM model is shown in Figure 9.

A hyper plane is used to express numerous classes in multidimensional space in an SVM model. In order to minimize the inaccuracy, SVM will generate the hyper plane repeatedly. The goal of SVM is to categorize datasets so that the biggest marginal hyper plane can be found (MMH). The data points that are closest to the hyper plane are called support vectors. As indicated in the diagram above, these data points will be utilized to define a distinct line. A hyper plane is a decision plane or space that is divided into several object types. The distance between two lines drawn on the nearest data points belonging to separate groups can be described as the margin. It is the distance between the line and the support vectors that is perpendicular to each other. A high margin is considered a positive margin, whereas a small margin is regarded as a negative margin.

#### 2.3.6. Voting Classifier

A voting classifier is a kind of ML model that trains on an ensemble of several models and predicts an output (class) based on the class with the highest probability of being chosen as the output [42].  Figure 10 depicts the voting classifier model's flowchart.

Voting encapsulates the technique that we will use to assess different training models. There are two ways to vote:

- Soft voting: This step sums and averages the projected probability vectors for each model. The class with the greatest value is declared the winner and outputted. While this seems to be a reasonable and logical approach, it is only advised if the individual classifiers are properly calibrated. This technique is similar to calculating the weighted average of a collection of values, except that each of the different models contributes proportionately to the resulting output vector
- Hard voting: In this step, the classification outputs of all the different models are merged, and the mode value of the resulting output is specified as the final output value. Because the specific probability values of each model are ignored, this method is similar to calculating the arithmetic average of a given collection of values. Only the output of each model is considered

### 2.4. Matrices of Evaluation

Figure 11 depicts the diagram of the confusion matrix. Confusion matrixes are used to evaluate the performance of ML classification models. The confusion matrix was used to evaluate the performance of all models generated. The confusion matrix indicates how often our models properly forecast and how frequently they guess incorrectly. False positives and false negatives were allocated to badly predicted values, while true positives and true negatives were assigned to properly anticipated values. After organizing all of the predicted values in the matrix, the accuracy, precision-recall trade-off, and AUC of the model were utilized to evaluate its performance.

## 3. Result and Data Analysis

This section examines the models' ability, model predictions, inquiry, and ultimate results.

### 3.1. Data Visualization

A histogram is a graphical depiction of an infinite class recurrence dispersion. It is an area outline composed of square shapes with bases at the intervals between class borders and regions proportionate to the comparing classes' frequencies. Because the base fills in the spaces between class borders, such representations link all of the square shapes. Square forms have statures proportional to their comparable classes' frequencies, and their statures will correspond to the appropriate recurrence densities for various classes.  Figure 12 shows the histogram for the whole dataset. A histogram is used to depict the dataset's proportions.

Figure 12 shows that the maximum baseline value is 500, fetal movement is greater than 2000, uterine contractions are higher than 400, and other important features are distribution.

### 3.2. Visualization of Feature Selection

Figure 13 shows the visualization of the feature selection method. The feature selection helps to understand how the features are correlated with each other.

Figure 13 shows that the main target feature “diagnosis” is positively corelated with fractal_dimension_mean, texure_se, smoothness_se, symmetry_se, and fractal_dimension_se. The rest of the features are negatively correlated with the target feature (diagnosis). The fetal health is 15% related to the baseline value. It has a 13% positive correlation with severe decelerations. However, it has the highest correlation with prolonged decelerations, which is 48%.

### 3.3. Accuracy of the Model

#### 3.3.1. Random Forest

Figure 14 shows the random forest model's classification report.

Here, the overall achieved F1-score is 98%. The individual F1-score is 97% for normal, 97% for suspected, and 99% for pathological.  Figure 15 shows the OOB error vs n_trees graph for the random forest classifier. From this, we can see that the error percentage is decreasing with the increase in the number of trees. The highest number of trees in this case is 400.

Figure 16 displays the prediction of the random forest model. The projected result is displayed in the confusion matrix, as well as the model's computed performance. The total number of correct predictions is 1453, with 37 incorrect forecasts.

#### 3.3.2. Decision Tree

Figure 17 shows the DT model's classification report. Here, the overall achieved F1-score is 96%. The individual F1-score is 95% for normal, 94% for suspected, and 98% for pathological.  Figure 18 displays the prediction of the DT model. The projected result is displayed in the confusion matrix, as well as the model's computed performance. The total number of correct predictions is 1426, with 64 incorrect forecasts.

#### 3.3.3. K-Nearest Neighbor

Figure 19 shows the K-nearest neighbor model's classification report. Here, the overall achieved F1-score is 90%. The individual F1-score is 89% for normal, 87% for suspected, and 94% for pathological.  Figure 20 displays the prediction of the KNN. The projected result is displayed in the confusion matrix, as well as the model's computed performance. The total number of correct predictions is 1344, with 146 incorrect forecasts.

#### 3.3.4. Logistic Regression

Figure 21 shows the LR model's classification report. Here, the overall achieved F1-score is 96%. The individual F1-score is 95% for normal, 94% for suspected, and 99% for pathological.  Figure 22 displays the prediction of the DT. The projected result is displayed in the confusion matrix, as well as the model's computed performance. The total number of correct predictions is 1431, with 59 incorrect forecasts.

#### 3.3.5. Support Vector Machine

Figure 23 shows the SVM model's classification report. Here, the overall achieved F1-score is 97%. The individual F1-score is 96% for normal, 95% for suspected, and 99% for pathological.  Figure 24 displays the prediction of the SVM model. The projected result is displayed in the confusion matrix, as well as the model's computed performance. The total number of correct predictions is 1439, with 51 incorrect forecasts.

#### 3.3.6. Voting Classifier

Figure 25 shows the voting classification model's classification report. Here, the overall achieved F1-score is 97%. The individual F1-score is 97% for normal, 96% for suspected, and 99% for pathological.  Figure 26 displays the prediction of the voting classifier model. The projected result is displayed in the confusion matrix, as well as the model's computed performance. The total number of correct predictions is 1452, with 38 incorrect forecasts.

### 3.4. Model Comparison

Table 1 compares the models to those in previous research papers. The table clearly shows that among the many models in the framework, RF is the best. It has a higher F1-score and has greater exactness, review, and the region beneath the bend.

The decision tree achieved 96% accuracy in this paper, but in [24], they achieved only 86% accuracy by using the same model. The accuracy rate of decision trees and logistic regression is the same. KNN achieved the lowest accuracy of 90 percent.

## 4. Conclusion

CTG data is useful for obstetricians since it allows them to detect fetal anomalies and decide on medical intervention before the infant sustains permanent harm. However, the obstetrician's visual interpretation of the CTG data may not be impartial or accurate. The use of decision support systems in medicine to identify and anticipate aberrant conditions is becoming an increasingly popular trend. We utilized CTG data to concentrate on the diagnosis of prenatal hazards in this research. Thus, utilizing the CTG dataset, ML models may be used as a decision support system to detect prenatal anomalies. On the other hand, we used several well-known ML methods in our research. The random forest, decision tree, K-nearest neighbor, voting classifier, support vector classifier, and logistic regression were the most accurate algorithms, with 97.51 percent, 95.70 percent, 90.20 percent, 97.45 percent, 96.57 percent, and 96.04 percent accuracy, respectively. The accuracy percentage of the models used in this research is much greater than that of previous investigations, suggesting that the models used in this investigation are more trustworthy. Numerous model comparisons have shown their robustness, and the scheme may be deduced from the research analysis. In the future, different complicated machine learning models can be implemented to make this system more robust.

## Figures and Tables

**Figure 1:** Total number of normal (1), suspect (2), and pathological (3) data.

**Figure 2:** Percentage of normal, suspect, and pathological data.

**Figure 3:** Total number of normal (1), suspect (2), and pathological (3) data after balancing.

**Figure 4:** System architectural diagram.

**Figure 5:** Flowchart of Random Forest Classifier.

**Figure 6:** Flowchart of decision tree classifier.

**Figure 7:** Flowchart of K-NN classifier.

**Figure 8:** Flowchart of logistic regression classifier.

**Figure 9:** Flowchart of support vector machine classifier.

**Figure 10:** Flowchart of voting classifier.

**Figure 11:** Diagram of confusion matrix.

**Figure 12:** Histogram of the dataset.

**Figure 13:** Visualization of feature selection.

**Figure 14:** Random Forest Model's classification report.

**Figure 15:** OOB error vs n_trees.

**Figure 16:** Random forest confusion matrix.

**Figure 17:** Decision tree model's classification report.

**Figure 18:** Decision tree confusion matrix.

**Figure 19:** KNN classification report.

**Figure 20:** KNN confusion matrix.

**Figure 21:** Logistic regression classification report.

**Figure 22:** Logistic regression confusion matrix.

**Figure 23:** SVM classification report.

**Figure 24:** SVM confusion matrix.

**Figure 25:** Voting classifier classification report.

**Figure 26:** Voting classifier confusion matrix.

**Table 1:** Model comparison.

This paper (model name)	Accuracy (%)	Reference paper (model name)	Accuracy (%)
Random forest	98	Ref [24] Discriminant Analysis	82.1
Decision tree	96	Ref [24] Decision Tree	86
K-nearest neighbor	90	Ref [16] SVM	84
Logistic regression	96	Ref [16] Naïve Bayes	83.7

## Data Availability

The data utilized to support this research findings is accessible online at http://archive.ics.uci.edu/ml/datasets/Cardiotocography.
